# Joint detection of *ERCC1*, *TUBB3*, and *TYMS* guidance selection of docetaxel, 5-fluorouracil and cisplatin (DDP) individual chemotherapy in advanced gastric cancer patients

This article has been retracted.

**DOI:** 10.1186/s40001-014-0050-z

**Published:** 2014-09-16

**Authors:** Yushuang Luo, Zhanquan Li, Sen Cui, Cunfang Shen, Junhui Zhao, Milu Wu, Yuying Li, Miaozhou Wang, Rong Chen, Zhibo Liu, Ge Ri-li

**Affiliations:** Affiliated Hospital of Qinghai University, Kunlong Road 16, Tongren Road 29, Xining, 810001 China; Research Center for High Altitude Medicine, Qinghai University Medical School of Medicne, Qinghai, 810001 China

**Keywords:** Gastric cancer, ERCC1, TUBB3, TYMS, Chemotherapy

## Abstract

**Background:**

To investigate the guidance selection of docetaxel (D), cisplatin (DDP) (C), and 5-fluorouracil (5-FU) (F) as individual chemotherapy agents via joint detection of *ERCC1*, *TUBB3*, and *TYMS* genes in patients with advanced gastric cancer (AGC).

**Method:**

Clinical data of 120 patients with AGC who enrolled in our hospital between May 2009 and May 2012 were analyzed. These patients were randomly assigned to experimental and control groups. The mRNA expression of *ERCC1*, *TUBB3*, and *TYMS* was measured by DNA chip technology in the experimental group. Different chemotherapies were administered according to the mRNA expression levels of the three genes, while DCF chemotherapy was directly applied to the control group. Correlation between the three genes’ mRNA levels, efficiency rate, the median time to progression (MTP), median survival time (MST) and adverse reactions was evaluated.

**Results:**

As a result, there was a significant correlation between *ERCC1* and *TUBB3* mRNA expression (*P* = 0.005), but no obvious correlation between *TUBB3* and *TYMS* or *ERCC1* and *TYMS*. There was also no significant difference in the efficiency rate of chemotherapy (50% versus 55%; *P* = 0.357) and the MTP (10 months versus 7 months; *P* = 0.091) between the two groups. However, there was obvious significance in MST (13.7 months versus 11.6 months; *P* = 0.004). Additionally, the experimental group provided us with a more effective way for controlling adverse reactions to chemotherapy.

**Conclusion:**

Combination regimen of D, C, and F in AGC patients according to their *ERCC1*, *TUBB3*, and *TYMS* mRNA expression level may reduce adverse reactions and improve MST.

## Background

Gastric cancer, which ranks as the cancer with the second highest mortality rate, is the fourth most common malignant tumor overall [1]. The incidence and mortality of gastric cancer is high in China, especially in Qinghai province. However, most newly diagnosed patients tend to be in the late stages [2-4]. At present, systemic chemotherapy is the main treatment option for these patients [5-7]. However, the effectiveness of chemotherapy in advanced gastric cancer (AGC) is less than 50%, and these patients have a median survival time (MST) of six to nine months, rarely exceed one year [8]. Although many chemotherapy regimens in randomized studies have been examined, there is no international standard for gastric cancer treatment [5,9]. Previous reports have shown that therapy using docetaxel and cisplatin (DPP) plus fluorouracil (5-FU) improved survival of patients with advanced cancer, but the clinical application was limited due to the toxicity [10].

The development of human genomics, pharmacogenomics, and tumor molecular biology shows a unique genetic map [11]. The genetic differences relating to drug sensitivity and resistance in patients have been found by detecting genetic alterations in patients using pharmacogenomics [12]. Subsequently, selection of appropriate chemotherapeutic drugs will be benefited leading to efficacy improvement, reducing side effects, and avoiding ineffective treatment. Chemotherapeutic tolerance and drug resistance are the main causes of chemotherapy failure in gastric cancer [13].

A number of drug-related genetic factors include 5-FU metabolism-associated genes (for example, thymidylate synthase (*TYMS*), deoxythymidylate kinase (*DTYMK*)) [14], taxol-related genes (Class III β-tubulin (*TUBB3*)) [15], and platinum-related genes (for example, excision repair cross-complementation group (*ERCC1*) and breast cancer 1, early onset (*BRCA1*)) [16]. *ERCC1* group participates in drug resistance in the response to platinum-based chemotherapy [17]. Its mRNA expression level has shown a negative correlation with platinum-based cancer chemotherapy and survival [18]. Sensitivity to platinum-based chemotherapy has been observed in patients with low *ERCC1* expression, while resistance has been noted in whose with high expression level [19,20]. The patients with tumors of high *TUBB3* mRNA expression present with poorer treatment outcomes with shorter MST on chemotherapy with anti-microtubule drugs and *vice versa* [21,22]. *TYMS* encodes the rate-limiting enzyme thymidylate synthase (TS), which is responsible for pyrimidine nucleotide synthesis and tumor growth [23]. TS is also the target enzyme for 5-FU to exert its cytotoxic effects [24]. The tumor patients with low *TYMS* mRNA levels showed a better response with longer MST on fluorine-based chemotherapy. Through meta-analysis, Hu *et al*. [25] have pointed out that *TYMS* is one of the useful predictive and prognostic genetic factors.

Tumor drug resistance is controlled by a complex web of gene networks. It has been observed that there are obvious limitations to testing a single target gene. Predication of clinical drug efficacy for patients can be achieved by detecting the expression pattern of a single gene or marker [26]. Therefore, it is important to screen drugs for patients by means of detecting target genes. With the development of individualized treatment and molecular detection, it is now possible for parallel determination of target genes.

In recent years, some studies have been performed to identify biomarkers along with clinical outcomes as the individual chemotherapy for AGC; this may improve treatment efficacy and avoid unnecessary side effects. However, few studies have indicated the efficiency of individual chemotherapy for AGC by detecting the mRNA expression level of genes to guide the selection of specific drugs. To elucidate more insights into individual chemotherapy for AGC, we investigated the guidance selection of docetaxel (D), DDP (C), and 5-FU (F) as individual chemotherapy via joint detection of *ERCC1*, *TUBB3*, and *TYMS* genes. The results of this investigation might contribute to guiding therapy for chemotherapy selection in patients with AGC.

## Methods

### Patient selection

Patients with AGC according to histopathology were selected from the Department of Tumor, Internal Medicine Affiliated Hospital of Qinghai University between May 2009 and May 2012. One hundred and twenty patients aged 21 to 70 years old (28 patients in the ≤ 35-year-old group; 92 patients in the 36- to 70-year-old age group; median age was 59 years old) including 85 males and 35 females, were chosen for further investigation. The baseline clinical characteristics are shown in Table 1 based on American Joint Committee on Cancer (AJCC) TNM staging system (2010) [27]. The inclusion criteria were as follows: patients with AGC presenting a measurable primary lesion, diameter ≥ 20 mm, chest radiograph showing ≥ 20 mm, magnetic resonance imaging (MRI) (3.0 T) showing ≥ 10 mm or computed tomography (CT) (256-slice) showed ≥ 10 mm; survival estimates of Eastern Cooperative Oncology Group (ECOG) ≤ 2 that have a median survival of more than 3 months; patients with normal peripheral blood count, no major organ damage, normal ECG, no non-healing wounds. Patient participation was voluntary and required signed informed written consent.

**Table 1:** **Baseline clinical characteristics of the two advanced gastric cancer patient groups before chemotherapy**

**Item**	**Number of patients**	**Experimental group**	**Control group**	***P***
Gender	120	60	60	
Male	85	42	43	1
Female	35	18	17	
Age				
≤ 35	28	13	15	0.829
36 to 70	92	47	45	
Phase				
III C	42	22	20	0.848
IV	78	38	40	
Tumor location				
Proximal stomach	28	15	13	1
Gastric body	40	18	22	
Distal stomach	52	27	25	
ECOG score				
0 to 1	46	24	22	0.851
2	74	36	38	
Pathological type				
Well differentiated	16	7	9	0.8
Moderately differentiated	28	15	13	
Poorly differentiated	76	38	38	

Patient exclusion criteria were as follows: pregnancy, breast-feeding and female patients of childbearing age not using contraception; uncontrolled acute infection; suppuration, chronic wound infection, and delayed wound healing; patients with serious heart disease; neurological disorder and mental illness; undifferentiated carcinoma and squamous cell carcinoma.

The exit criteria were as follows: cases of severe drug-related toxicity; inability to tolerate side effects; patients withdrawing from the study; patients who researchers believe should be withdrawn.

The enrolled patients with AGC in our study were randomly assigned to two groups: the experimental group and the control group. The mRNA expression of *ERCC1*, *TUBB3*, and *TYMS* were measured by DNA chip technology in the experimental group. Then, the experimental group was divided into four subgroups according to the mRNA expression of the three genes: low expression of a single-gene subgroup, low expression of double-gene subgroup, low expression of triple-gene subgroup, and non-low expression of triple-gene subgroup.

### Gene expression detection

DNA chip technology was used to investigate the expression patterns of genes based on hybridization of labeled RNA probes [28]. To elucidate the mRNA levels of *ERCC1*, *TUBB3*, and *TYMS* in gastric cancer tissue, the DNA chip technology was employed as described by Liu *et al*. [29]. Firstly, total RNA was released from gastric carcinoma in formalin-fixed paraffin-embedded tissue. The targeted mRNA probe was bound to the microsphere. Target and signal amplification was then performed by hybridization reaction. Finally, the processed mRNA probe were combined with streptavidin-phycoerythrin (SA-PE) and analyzed by a Luminex 100 flow cytometer (Luminex Corp., Austin, TX, USA). p2-microglobulin, transferrin receptor, and TATA-box binding protein were used as controls for housekeeping gene expression. The mean fluorescence intensity (MFI) values of the background were subtracted from the MFI values of the sample to determine the net MFI, which represents the relative mRNA expressions of *ERCC1*, *TUBB3*, and *TYMS*.

To estimate these three gene expression patterns in patients over the whole distribution, the quartile method was used. In this method, a percentage rate less than 37.5% denotes lower expression; from 37.5% to 62.5% denotes mid-level expression, while more than 62.5% denotes higher expression.

### Chemotherapy regimens

The chemotherapy regimen comprising D, C and F was administered to low (or mid-level) expression of *ERCC1*, *TUBB3*, and *TYMS* patients respectively in the experiment group. D, C, and F combination chemotherapy was utilized for fourteen cases (low (or mid-level) expression of *ERCC1*, *TUBB3* and *TUBB3*); in pair-wise fashion, D plus C was administered to seventeen cases (low (or mid-level) expression of *ERCC1* and *TUBB3*); D plus F was administered to ten cases (low (or mid-level) expression of *TUBB3* and *TYMS*); C combined with F therapy was used for eight cases (low (or mid-level) expression of *ERCC1* and *TYMS*); isolated D, C, and F were given to six, three, and two cases, respectively. The doses of D, C, and F in the chemotherapy regimes were 75 mg/m^2^, 75 mg/m^2^, and 750 mg/m^2^, respectively. The control-group patients were given the combination chemotherapy of D, C, and F (at same dose levels as the experiment groups). The efficacy was tested for two periods of 21 days.

### Evaluation of efficacy and indicator in patients

Short-term clinical effects in patients with solid tumors were classified into complete response (CR), partial response (PR), stable disease, and progressive disease (PD) according to Response Evaluation Criteria in Solid Tumors (RECIST) 1.1. CR and PR represent the effective influence on patients, while PD represents the ineffective impact on patients. Adverse reactions were divided into grades 0 to IV based on National Cancer Institute Common Toxicity Criteria, version 3.0 (NCI-CTC 3.0). The indices relating to patients’ survival were identified as time to progression and overall survival time. Patient follow-up was once every two months via telephone calls after stopping treatment up until death.

### Statistical method

Data were analyzed using SPSS software program version 17.0 (SPSS Inc., Chicago, IL, USA). The χ^2^ and Fisher’s exact tests were carried out for count data. Exact calculation of the R × C table used Monte Carlo. The rank correlation test was then computed to reveal the correlation between groups. The Kaplan-Meier analysis provided survival estimates and the log-rank test was used to compare survival curves for patients between groups. Cox regression model analysis of factors potentially related to survival was used to identify the independent factors that may significantly affect survival. A two-sided test (α = 0.05) was performed for all statistical tests.

## Results

### Correlation of *ERCC1*, *TUBB3*, and *TYMS* mRNA levels in patients

To investigate the *ERCC1*, *TUBB3*, and *TYMS* mRNA expression of patients in the experimental group, DNA chip technology was performed. Results revealed that 36 (60.00%) and 16 (26.67%) patients showed low and mid-level *ERCC1* levels respectively. Thirty-three (55.00%) and 15 (25.00%) patients were shown to have low and mid-levels respectively of *TUBB3* mRNA expression. Twenty-seven (45.00%) and 15 (25.00%) patients yielded low and mid-levels of *TYMS* mRNA. There were 18 (30.00%), 27 (45.00%), and 10 (16.67%) cases showing low expression of single, double, and triple genes, respectively. However, there were eight cases that showed high or mid-level but not low expression of these three genes.

Rank correlation methods were then computed to identify the relationship between *ERCC1*, *TUBB3*, and *TYMS* mRNA levels in all patients. As a result, there was a poorly-correlated relationship between the mRNA levels of *ERCC1* and *TUBB3* (γ = 0.361, *P* = 0.005). Nevertheless, this phenomenon was not observed in mRNA levels of *TUBB3* and *TYMS*, or between *ERCC1* and *TYMS* (*P* > 0.05).

### Effectiveness of chemotherapy

Total effective rate of chemotherapy in 120 patients with AGC was 52.50% (63/120). The chemotherapy showed 50.00% (30/60) and 55.00% (33/60) effectiveness rates in the experiment group and control group, respectively. However, despite small differences in chemotherapy effectiveness rate for the two groups, no significant difference was observed (χ^2^ = 0.301, *P* = 0.357).

We then proposed an exact Monte Carlo approach to reveal the chemotherapy response among four subgroups of the experiment group (*P* = 0.002). As shown in Table 2, the results indicated that no obvious difference was found between the single-gene subgroup (low-level expression) and those subgroups of the double gene (low-level expression) and non-low expression of triple gene (*P* = 0.721, *P* = 0.084, respectively). However, there was a significant difference between the low expression of a single gene and the low expression of triple gene (*P* = 0.025). The double-gene subgroup with low or mid-level expression pattern significantly improved with chemotherapy compared with the triple-gene subgroup with low or mid-level expression (*P* = 0.001). The triple-gene subgroup with low or mid-level expression also significantly improved chemotherapeutic effectiveness in comparison with non-low expression of triple gene (*P* < 0.001**)**.

**Table 2:** **Comparison of therapeutic efficacy among experimental subgroups**

**Subgroups**	**Number of patients**	**Effective number of patients**	**Efficient rate (%)**
Low expression of single gene	18	10	55.6^bcd^
Low expression of double gene	24	12	50^acd^
Low expression of triple gene	10	10	100^abd^
Non-low expression of triple gene	8	1	12.5^abc^

*P* = 0.721 (a compared with b); *P* = 0.025 (a compared with c); *P* = 0.084 (a compared with d); *P* = 0.101 (b compared with c); *P* = 0.006 (b compared with d); *P* < 0.001 (c compared with d).

### The MTP assay

As shown in Figure 1, median time to progression (MTP) was analyzed to study the chemotherapeutic effect between the two groups. The results showed that the MTP was 9 months for the 120 patients. In addition, the MTP was ten months and seven months for the experiment group and the control group, respectively. The log-rank test demonstrated that there was no significant difference between the two groups (χ^2^ = 2.849, *P* = 0.091).

**Figure 1:** **Kaplan-Meier survival curves for time to progression in patients with advanced gastric cancer.**

### The MST assay

As shown in Figure 2, the MST was then analyzed for all patients with AGC. A 12-month MST was observed in 120 patients. The MST of the experimental group was 13.7 months, while for the control group was only 11.6 months. A statistically significant difference was observed between the two groups (χ^2^ = 8.310, *P* = 0.004). The result also showed that the experimental group had a longer survival curve compared to the control group. However, no significant difference in MST was found between the four subgroups of the experiment group.

**Figure 2:** **The median survival curves of the patients with advanced gastric cancer.**

### Comparison of adverse reactions

We observed that the types of adverse reaction were similar in all 120 patients with AGC. The types of adverse reaction included hematologic toxicity, gastrointestinal reactions, neurotoxicity, and liver and kidney dysfunction. Hematologic toxicity includes leukopenia, decrease in hemoglobin, and thrombocytopenia. The patients in the experimental group experienced hematologic toxicity of a grade 1 to 2, which was better than the control group which experienced grade 3 to 4. There was a significant difference in hematologic toxicity between the two groups (*P* = 0.048, *P* = 0.016, *P* < 0.001). Gastrointestinal reactions exhibited included nausea, vomiting, and diarrhea. The patients in the control group experienced gastrointestinal reactions of a grade 3 to 4, worse than the experimental group (*P* < 0.001, *P* = 0.041). The experimental group also performed better regarding peripheral neurotoxicity, liver damage, and kidney damage than the control group (*P* = 0.01, *P* = 0.01, *P* = 0.01). There were no deaths in the two groups relating to chemotherapy, but eight cases were withdrawn due to adverse reactions to chemotherapy in the control group compared with one in the experimental group. Thus, compared with the control group, the experimental group demonstrated a more effective way for controlling adverse reactions from chemotherapy for AGC patients.

## Discussion

In this present study, 120 patients with AGC were enrolled and then randomly assigned to experimental and control groups. Different chemotherapy regimens (DCF, DC, CF, DF, D, C and F chemotherapies) were administrated to 60 patients with AGC based on analysis test data of *ERCC1*, *TUBB3*, and *TYMS* mRNA expression levels in the experimental group. Meanwhile, the other 60 patients with AGC directly received the DCF chemotherapy regimen. Then, we evaluated the correlation between the three genes’ mRNA levels, efficiency rate, MTP, MST and adverse reactions. The results showed that there was a significant correlation between *ERCC1* and *TUBB3* mRNA expression levels, but no obvious correlation between *TUBB3* and *TYMS* or *ERCC1* and *TYMS*. Also, there was no significant difference in the efficiency rate of chemotherapy and MTP between the two groups. However, there was an obvious significant difference in MST. Additionally, the experimental group demonstrated a more effective way for controlling adverse reactions from chemotherapy.

An effective chemotherapy regimen is critical for AGC [30]. Our results showed that the chemotherapy effectiveness was 50% (experimental group) in the DCF program, or their combination. The rate is higher than a phase III study from the V-325 group and also higher than the research which involved 48 cases with DCF regimen palliative chemotherapy conducted by Huang *et al.* [21,31]. In our study, individualized chemotherapy was used in AGC patients according to their mRNA expression level of *ERCC1*, *TUBB3*, and *TYMS*, which may account for the higher rate. Besides, lower therapeutic effect in the V-325 study group may be influenced by the presence of more liver metastases or small sample size in phase III. The response to DCF regimens may also be affected by the number of chemotherapy cycles given to patients; a consideration that warrants further investigation.

This study found that a better response to chemotherapy occurs in *TUBB3*, *TYMS*, or *ERCC1* low-expression subgroups compared with mid- or high-expression groups, which is basically similar to conclusions drawn by Huang *et al*. [21] and Lu *et al*. [31]. Serious chemotherapeutic side effects, especially hematological toxicity, were observed in the DCF-treated patients, which is similar to the V-325 study reported by Ajani *et al*. [32]. We can conclude that DCF chemotherapy is effective, but with more side effects, in the treatment of AGC. Lower adverse reaction rates with good curative effect were shown in early stages under chemotherapy regimen selection based on *TUBB3*, *TYMS*, and *ERCC1* mRNA expression levels in gastric cancer patients.

This investigation showed that the MST and MTP was 11.6 and 7 months in the control group, which was extended by 1.4 months in the V-325 study group, respectively. Our results are consistent with a treatment effect that has been reported by Hu *et al*. [25]. Shorter survival in the V-325 study group may be due to the inclusion of more patients with liver metastases and fewer stage III patients. There was no significant difference in MTP between the experimental group and the control group, but the MST was significantly longer in the experimental group. This suggested that the chemotherapeutic drug extended the MST according to the expression of target genes. Previous reports showed the MST to be longer in patients with none or one resistance gene than in patients with more than two resistance genes [12]. In this study, there was no obvious difference among the four experimental subgroups. However, the small sample size here may influence the MST and a larger sample size will need to be evaluated.

## Conclusions

In conclusion, our study demonstrated that the combination regimen of D, C, and F in AGC patients according to their *ERCC1*, *TUBB3*, and *TYMS* mRNA expression level might reduce severe adverse reactions and improve the MST. However, further investigation and a larger clinical research sample are needed to further explore the application of multiple genetic targets to chemotherapy for patients with AGC.

## Abbreviations

5-FU: 5-fluorouracil
AGC: advanced gastric cancer
AJCC: American Joint Committee on Cancer
CR: complete response
CT: computed tomography
DPP: cisplatin
ECOG: Eastern Cooperative Oncology Group
MFI: mean fluorescence intensity
MRI: magnetic resonance imaging
MST: median survival time
NCI-CTC: National Cancer Institute Common Toxicity Criteria
MTP: median time to progression
PD: progressive disease
PR: partial response
RECIST: Response Evaluation Criteria in Solid Tumors
SA-PE: streptavidin-phycoerythrin
TS: thymidylate synthase
